RETRACTED

# Study of Nursing Models by Machine Learning in Children with Congenital Esophageal Atresia

**DOI:** 10.1155/2022/4147217

**Published:** 2022-04-10

**Authors:** Yu Zhang, Xueqiang Sun, Jingyun Shi, Zhenjuan Xiao

**Affiliations:** ^1^Neonatal Intensive Care Center, Gansu Provincial Maternity and Child-care Hospital, Lanzhou730050, Gansu, China; ^2^Department of Pediatric Surgery, The First Hospital of Lanzhou University.Lanzhou730000, Gansu, China

## Abstract

This research paper elucidates the clinical effect of an integrated nursing model of medical care and patient in the diagnosis and treatment of congenital esophageal atresia (CEA). For this purpose, a total of 120 children with CEA were selected as study subjects who were admitted to our hospital (January 2017 to April 2020). They were randomly divided into the control group and observation group. Each group had 60 cases. The control group was given routine nursing, while the observation group adopted the integrated nursing model of medical care. The integrated nursing model had the characteristics of recognizing and managing the CEA quickly and efficiently. Thus, it can help increase the survival rate of infants. This model works along with the parents to provide specialized services to the child. They were tasked to carefully observe the infants as well as calm the parents. They were also given the additional task of keeping track of patients who were currently admitted in the hospital and those who were already discharged. The tracking and communication were done with the help of a communication platform which is WeChat. The rehospitalization rate, 1-hour visit rate, accuracy rate of children with suspected postoperative complications, psychological status of children's parents, medical compliance, and satisfaction were compared between the two groups. The rehospitalization rate in the observation group was lower than that in the control group (*P* < 0.05). The 1-hour visit rate and accuracy of children with suspected postoperative complications in the observation group were higher than those in the control group (*P* < 0.05). The anxiety and depression scores of the parents in the observation group were lower than those in the control group (*P* < 0.05). The compliance and satisfaction of parents in the observation group were higher than those in the control group (*P* < 0.05). The clinical effect of the integrated nursing model of medical care and patient in CEA was highly satisfactory. It reduces the rehospitalization rate and enables timely diagnosis and treatment of suspicious complications effectively. It also improved parents' negative psychological emotions, compliance, and satisfaction.

RETRACTED

## 1. Introduction

Congenital esophageal atresia (CEA) is a birth defect in infants in which the esophagus is not linked to the stomach. This causes choking and breathing problems in the babies. It is a common disease in neonatal surgery. For this disease, surgery is the only preferable treatment. In recent years, with the development of multidisciplinary management, the level of treatment of CEA has improved significantly. The cure rate of CEA without serious cardiac malformations is over 90% [1]. The complications after CEA are not always the same. They range between 30% and 50%. It includes esophageal anastomotic stricture, anastomotic fistula, tracheoesophageal fistula recurrence, gastroesophageal reflux, tracheal softening, respiratory disease, and abnormal esophageal function [2]. The recognition and management of CEA complications will affect the survival probability of infants and bring a serious psychological burden to the families of the infants [3, 4]. The concept of integrated medical-nursing-patient care is a relatively advanced care model, which is based on the concept that the family of the child is the core, and physicians and nursing staff work together to provide specialized services for the child. It will improve the parents' awareness of the disease, make them actively cooperate with the treatment, and establish a good doctor-patient relationship [5]. In this study, we observed the clinical application effect of the integrated medical-nursing-patient care model in 60 cases of children with CEA and compared it with the intervention effect of the conventional care model. The aim was to explore the application effect of the integrated medical-nursing-patient care model in children with CEA.

In addition to environmental factors, patients' medical conditions and the treatment they receive at the time of hospitalization are also factors that influence their admission to the hospital relative to their health. Many diseases, such as chronic diseases, have long treatment cycles or even require lifelong treatment. Repeated hospital admissions are often required during the course of treatment. Unplanned readmission refers to the situation where a patient is readmitted for the same disease or related diseases within a short period after being discharged from the hospital. It is a negative indicator commonly used to assess the quality of hospital care. A high readmission rate can increase the financial burden on patients and cause waste of healthcare resources [6]. In one study, the annual 30-day readmission rate in the United States exceeded 20%, and the resulting healthcare costs exceeded $20 billion [7]. The readmission rate is an important indicator of the quality of healthcare services. Hospitals can effectively reduce the readmission rate if they predict the readmission population in advance that may be at high risk and take interventions such as follow-up visits to patients. Since it is difficult for physicians to assess readmission risk directly due to the complexity of factors affecting readmission, the use of readmission identification models based on machine learning and data mining is important for early readmission interventions. Very few patients in real healthcare data are readmitted, resulting in an extremely unbalanced dataset for readmission risk prediction. Therefore, the prediction results of traditional classification models show very low prediction accuracy for positive samples. Most of the real-life data are unbalanced datasets, and how to design classification algorithms to maximize the balance between the classification accuracy of positive and negative samples has become a hot research topic in the field of machine learning.

RETRACTED

Population and individual health risk assessment are important for raising people's health awareness, optimizing hospital resource management, and improving medical processes. Nowadays, with the development of medical informatization, many medical assistance systems have come into being. Using the technical means related to data mining and machine learning, combined with the massive and rich medical data, we can build a health risk assessment system applicable to the population and individuals. It can not only help hospitals to be more forward-looking in their surgery process but also help patients understand more about their health condition through this system and take protective measures in advance.

The rest of the research paper is structured as follows. The next section will explain the related work done in this study. It will be followed by medical and nursing integration models. Next, the analysis of different cases will be discussed. After this, the case studies, discussion, and concluding remarks will be explained.

## 2. Related Work

Currently, healthcare integration still lacks a commonly accepted concept [2]. It argues that healthcare integration is about shared planning, decision making, goal setting and problem solving, and shared responsibility for patients. It requires mutual trust and respect from both participants [3]. It also argues that the concept of nurse-physician collaboration is more than just working together in a shared environment. It requires a common goal of providing quality care to solve patients' problems and shared responsibility for the patient. Interprofessional collaboration is a process in which each member of the healthcare team has specialized knowledge and skills that require interaction and collaboration between different healthcare professionals [4]. So far, different scholars still have different views on the concept of the healthcare integration model. Most of them encapsulate some common elements, namely, doctors and nurses respect and trust each other, form a closely collaborative treatment team, solve patients' problems together, improve clinical services, and improve the quality of treatment and care.

RETRACTED

## 3. Medical and Nursing Integration Models

In a survey of nine intensive care units, it was shown that nurse-physician cooperation helped reduce the occurrence of postoperative infections in critically ill patients. It shortened the treatment time and facilitated the recovery process of the patients [4]. Positive nurse-physician cooperation can improve nurses' job satisfaction, increase identification with the team, and reduce staff turnover [8]. It was observed that interprofessional teamwork between healthcare providers is essential to improve patient outcomes and quality of care, to develop and establish respectful interprofessional relationships between nurses and physicians, and to encourage continuing in-service training programs and workshops that focus on teamwork and communication [9]. The literature reports that inadequate collaboration and communication among healthcare professionals can negatively impact the delivery of healthcare and patient outcomes [10]. Since 2010, the West China Hospital of Sichuan University has put the integration model into clinical application, and then several hospitals in China have started to learn and explore it one after another [11]. It was found that the integrated clinical care model of medical and nursing care improved physicians' satisfaction. Nurses' self-confidence was also enhanced, and the attitude and feeling of cooperation between medical and nursing care were significantly improved through investigation [12]. It was concluded that medical and nursing cooperation in joint research work significantly increased the interest and motivation of medical and nursing staff in research. The number of published nursing research papers also increased significantly [6]. The implementation of the integrated medical and nursing management model to standardize the safe transfer of patients from ICU was found to significantly reduce the reentry rate and the incidence of transfer handover problems within 48 hours (*h*) after patients were transferred from ICU. It improved efficiency and reduced the occurrence of disputes between nurses and patients. The implementation of the integrated medical and nursing model is mainly through the establishment of integrated medical and nursing working groups, including joint medical and nursing room visits, joint health education, etc. It can better provide individualized, high-quality care for the patients. At present, domestic scholars are exploring based on learning and absorbing excellent experiences from abroad, and it is widely used in the nursing field and has achieved remarkable results.

RETRACTED

## 4. Analysis of the Effects of GAM Model on the Management of Patients with Congenital Esophageal Atresia (CEA)

Here, we will analyze different models used for the study and check if they can play a positive role for the patients. The details are as follows.

### 4.1. Model Construction

The GAM model can represent the independent variables in a summation form through a smoothing function. Therefore, it can be flexible in fitting nonlinear relationships. Since the number of daily hospitalizations obeys an over-discrete Poisson distribution, a GAM model with a semi-Poisson distribution (quasi-Poisson) as the link function is constructed. The model uses the number of disease admissions as the dependent variable, and the independent variable controls are as follows.

Nature spline (NS) and degrees of freedom (DF) are smoothing functions, which represent the long-term time trend and seasonal trend of daily admission.

Meteorological factors not only affect the concentration of air pollutants but also directly influence the number of daily hospital admissions. To assess the impact of meteorological factors on the estimation of pollutant effects in the GAM model, ns will be used to fit the mixed effects of meteorological factors, such as temperature (Temp), relative humidity (RH), rainfall (Rain), sunshine (Sun), and wind speed (Wind).

After controlling for confounding factors, the pollutants to be studied were added to the model to explore the effect of pollutants on the number of daily hospitalizations. The final model constructed can be expressed as

(1) $$\begin{array}{c} \log\left\{E\left(Y_{t}\right)\right\}=\alpha +\beta Z_{t-i}+ns\left(\text{Time},df=7*2\right)\\ +ns\left({\text{Temp}}_{06},df=3\right)+ns\left(RH_{0},df=3\right)\\ +ns\left({\text{Rain}}_{0},df=3\right)+ns\left({\text{Sun}}_{0},df=3\right)\\ +ns\left({\text{Wind }}_{0},df=3\right)+DOW_{t}+{\text{Holiday}}_{t}. \end{array}$$

### 4.2. Stratification Studies and Sensitivity Analysis

The sensitivity of the GAM model is divided into the following two aspects.

*Single-Day Lag*. The single-day lag at day (*t*) examines the effect of pollutants from day t-i to day t-1 on the number of hospitalizations at day *t*.

*Moving Average Lag*. It refers to the effect of moving average (lag0i) of day *t* and day t-i on the number of hospitalizations on day *t*. For example, lag01, lag02....

RETRACTED

In the study of this thesis, the lag effect is studied in the range of lag1-lag7, lag01-lag07.

Two pollutants were controlled as the main variables in the model to explore the effect of the influence of the two pollutants and whether the pollutants have independent health hazards.

### 4.3. Attention-LSTM Model

In this paper, we use the LSTM network to capture the trend of advertisement popularity and introduce the attention mechanism into the LSTM network. It helps reduce the interference of external factors and construct the attention-LSTM model based on the attention mechanism. By analyzing the feedback information of users' likes, views, comments, etc., given the time interval *t*, the amount of user feedback over time is constructed as a time series *d*_*i*_, and then the feedback series {*d*_1_, *d*_2_, ..., *d*_*i*_} is obtained. The calculation formula of the LSTM network is rewritten as

(2) $$\begin{array}{c} G_{t}^{i}=\sigma \left(W^{i}x_{t-1}+U^{i}c_{t-1}+D^{i}h_{t-1}+b^{i}\right),\\ G_{t}^{f}=\sigma \left(W^{f}x_{t-1}+U^{f}c_{t-1}+D^{f}h_{t-1}+b^{f}\right),\\ c_{t}=G_{t}^{f}hh_{t-1}+G_{t}^{i}*\;\tanh\left(W^{c}x_{t-1}+D^{c}h_{t-1}+b^{c}\right),\\ G_{t}^{{}^{\circ}}=\sigma \left(W^{0}x_{t-1}+U^{0}c_{t-1}+{}^{D^{{}^{\circ}}}h_{t-1}+{}^{b^{{}^{\circ}}}\right),\\ h_{t}=G_{t}^{0}*\;\tanh\left(c_{t}\right). \end{array}$$

The computation process of the attention-LSTM model is as follows.

Given a certain time interval *t*, the *n* hidden layer outputs are denoted as *H*_*i*_:

(3) $$\begin{array}{c} H_{i}=\left\{h_{1},h_{2},...,h_{n}\right\}. \end{array}$$

These hidden layers output *h*_*i*_ after the softmax layer to obtain the attention weights:

(4) $$\begin{array}{c} a_{i}=\text{softmax}{\left(h_{i}\right)}^{*}\left[\left(G_{t}^{{}^{\circ}}\right)*\tanh\left(c_{t}\right)\right]. \end{array}$$

Record the attention weight as *A*_*i*_：

(5) $$\begin{array}{c} A_{i}=\left(a_{1},a_{2},\cdots ,a_{n}\right). \end{array}$$

Then, the attention-LSTM model outputs the popular trend at this time：

(6) $$\begin{array}{c} O_{A-L}=a_{i}\left\{G_{t}^{0}*\;\tanh\left(c_{t}\right)\right\}. \end{array}$$

From the experimental results, the attention-LSTM model can effectively capture the popularity trend of advertisements， as shown in Figure 1. It is very helpful to improve the performance of the popularity prediction model [28].

### 4.4. NFM Model

The content of ads, including ad types and numerical information, usually provides useful information for popularity prediction and is one of the key factors affecting the popularity of ads. For different types of advertisements, different users have different preferences, and their feedback performance is very different [3], 29]. The NFM model combines linear second-order feature interactions and nonlinear higher-order feature interactions to learn features from sparse data. It effectively improves the feature representation capability.  Figure 2 shows the NFM model for content feature learning.

RETRACTED

For example, given the set of ad types as *M*=(*m*_1_, *m*_2_, ⋯, *m*_*k*_), for the *i* (*i* = 1, 2, ..., k) ad mi types, the one-hot feature vector *x* of the ad types is dimensioned down using the embedding technique to obtain the embedding vector representation of the video types:

(7) $$\begin{array}{c} \nu_{x}=\left\{x_{1}\lambda_{1},x_{2}\lambda_{2},\cdots ,x_{n}\lambda_{n}\right\}. \end{array}$$

Input the embedding vector *ν*_*x*_ to the second-order interaction layer:

(8) $$\begin{array}{c} z_{BI}\left(\nu_{x}\right)=\sum_{i=1}^{n}\sum_{j=i+1}^{n}x_{i}\lambda_{i}\Theta x_{j}\lambda_{j}, \end{array}$$

where Θ means (*λ*_*i*_Θ*λ*_*j*_)_*k*_=*λ*_*ik*_*λ*_*jk*_, and the second-order interaction layer is a pooling operation that converts the embedding matrix of text features into a vector. The output *z*_BI_(*ν*_*x*_) of the second-order interaction layer is input to the hidden layer and is computed as

(9) $$\begin{array}{c} \left\{\begin{array}{c} y_{1}=\sigma \left(W_{1}z_{BI}\left(\nu_{x}\right)+b_{1}\right),\\ y_{2}=\sigma \left(W_{2}y_{1}+b_{2}\right),\\ \vdots \\ y_{L}=\sigma \left(W_{L}y_{L-1}+b_{L}\right), \end{array}\right) \end{array}$$

where *σ*, *W*_*L*_, and *b*_*L*_ are the sigmoid function, the weight matrix, and bias vector of the hidden layer, respectively, and *L* is the number of layers of the hidden layer [30].

(10) $$\begin{array}{c} O_{NFM}=w_{0}+\sum_{i=1}^{n}w_{i}x_{i}+q^{T}\left(\text{softmax}\left(W_{L}y_{L-1}+b_{L}\right)\right). \end{array}$$

## 5. Case Study

The case studies of different subjects are explained as under.

### 5.1. General Information

One hundred and twenty children with type III congenital esophageal atresia admitted to our hospital (January 2017 to April 2020) were selected as the study subjects.

#### 5.1.1. Inclusion Criteria

The inclusion criteria include patients with

- Type III esophageal atresia.
- No chromosomal abnormalities.
- No serious precocious heart disease (except for arteriovenous ducts, patent foramen ovale, and small ventricular septal defect).
- No serious physical disease, no history of psychiatric disorders, and drug dependence in parents.
- Parents with elementary school education or above, able to read and understand the questions.

Family members were informed, and they signed an informed consent form to cooperate with this study. In this study, the children and families were randomly assigned in a 1 : 1 ratio into a control group and an observation group. Each group had 60 cases. The division was made with the help of a simple randomization method of the computer system. There was no statistically significant difference between the two groups in terms of gestational age, sex, birth weight, 1-minute Apgar score, parents' age, and education level (*p* > 0.05), and the differences were comparable, as shown in Table 1.

RETRACTED

On the one hand, we strengthen the communication among doctors, nurses, and patients through various ways to establish trust between doctors and patients and upload videos of the children through WeChat peer-to-peer, 2 to 3 times a week. Also, we increase the number of uploads appropriately according to the anxiety of the parents of the children, so that the parents can understand the health status of the children in time and relieve their anxiety. On the other hand, we strengthen professional care in many aspects and communicate with the doctors, including airway care, such as keeping the airway open, regular nebulization, back-patting, and sputum aspiration, and paying attention to not reaching the location of the tracheal fistula. In addition, in order to avoid complications, medical staff should carry out suction. The duty of the nurse is to take care of various pipes, such as gastric tube, thoracic drainage tube, deep vein, and other corresponding pipes, report any abnormalities to the doctor, and take good care of the patient's skin together with the doctor. The patient should turn over frequently to avoid pressure ulcer and hard swelling; closely monitor the child's condition, health and any vital signs.

### 5.2. Results

In both groups, children were revisited for fever, choking, laryngeal sounds, wounds, etc. For the number of revisits in the observation group, see Table 2.

The difference between the anxiety and depression scores of the parents of the two groups before the intervention was not statistically significant (*P* > 0.05). After the intervention, the SAS and SDS scores of the observation group were lower than those of the preintervention and control groups (*P* < 0.05), as shown in Table 3.

The compliance rate is shown in Table 4.

## 6. Experimental Results and Analysis

The experimental results and analysis of different study subjects are explained below.

### 6.1. Single-Pollutant Model Effect Results

The effects of the air pollutants *PM*_2.5_, *PM*_10_, *SO*_2_, *NO*_2_, CO, and *O*_3_ on the number of daily hospital admissions for respiratory, circulatory, and digestive diseases were analyzed according to the GAM model presented. The results are based on single pollutant results.

RETRACTED

Table 5 shows the effect of each pollutant on the number of hospitalizations for the three diseases in the single-pollutant model. It can be seen that all pollutants except O_3_ had significant effects on the number of respiratory hospitalizations (*p* < 0.05). 10 *μ*g increase in *PM*_2.5_, *PM*_10_, *SO*_2_, and *NO*_2_ pollutant concentrations caused 0.3%, 0.21%, 2.43%, and 1.17% increase in daily respiratory hospitalizations, respectively. The number of respiratory hospitalizations increased by 0.47% for each 0.1 mg increase in CO. The table also shows that a corresponding unit increase in *SO*_2_, *NO*_2_, and CO would increase the number of circulatory hospitalizations by 2.84%, 1.4%, and 0.6%, respectively. No effect of pollutants on the number of digestive system hospitalizations was found.

### 6.2. Hysteresis Effect Analysis

The results of the lag effect study based on the GAM model study are shown in Figures 3–5. In the study of the lag effect of respiratory diseases, except for *O*_3_, the single-day lag effect of all pollutants gradually decreased with the increase of lag days and mainly showed acute effects, and the statistically significant effects were concentrated in lag0-lag2. The moving average lag effect increased with the volatility of lag days, and there was a significant increase in the effect compared to the single-day lag effect.

In the lagged effect study of circulatory disease, *SO*_2_ and CO had more significant moving average lagged effects on older adults. The effect of pollutants on overall circulatory disease hospitalizations was concentrated in lag0.  Figure 5 depicts the effect of pollutants on the number of daily hospitalizations for digestive disease. Although no significant pollutant effects on daily digestive system hospitalizations were found in the single-pollutant study. In the lagged-effects study, all pollutants except *O*_3_ showed significant lagged effects on the number of digestive system disease hospitalizations in children, mainly in lag5-lag7 and lag06-lag07.

## 7. Discussion

The integrated medical, nursing, and patient model is a family-centered service concept, and a new trinity of medical, nursing, and parents is reestablished through the Internet communication platform such as WeChat. It is a rapidly developing and advanced nursing concept that has been widely used in the management of various disciplines and systems of internal and external gynecological and pediatric diseases [9].

The results of this study showed that the readmission rate of children in the observation group was lower than that in the control group (*p* < 0.05). The 1-hour consultation and accuracy rates of suspected postoperative complications were higher than those in the control group (*p* < 0.05). This indicates that the readmission rate in the control group increased due to the lack of out-of-hospital home care after discharge, such as inappropriate feeding leading to aspiration pneumonia, while in the observation group, the medical and nursing staff provided professional guidance effectively through WeChat and other Internet methods. It improved the knowledge of the child's family about CEA and reduced the corresponding postoperative complications and also reduced the anxiety of parents due to repeated communication through the WeChat platform. At the same time, the repeated communication through the WeChat platform has reduced the number of visits to the hospital and the readmission rate due to parental anxiety, effectively reducing the burden on the child's family. For suspected postoperative complications, which may lead to poor prognosis if not treated in a timely manner, the observation group achieved early detection, green channel consultation, and timely treatment intervention through effective management and communication, which effectively improved the admission rate of children with suspected postoperative complications and thus improved the prognosis. This indicates that the integrated medical-nursing-patient model plays an important role in the management of CEA, which not only improves the prognosis of children but also increases parents' correct knowledge of the disease, improves parental cooperation, improves home care, and further improves the prognosis of children.

RETRACTED

CEA not only affects the health of the child but also puts a heavy psychological burden and financial pressure on the parents of the child. Parents of children with CEA often experience self-blame and guilt when faced with the possibility of postpartum depression and congenital disease and are prone to anxiety and depression due to financial pressure and lack of awareness of the disease. The results of this study showed that the parents of the children were mildly depressed and moderately anxious at the time of admission. The results suggest that medical and nursing staff should pay attention to the adverse psychological state of the child's family members while paying attention to the treatment and care of the child's condition and help the parents eliminate the adverse emotions through timely detection of the parents' adverse emotions and targeted interventions. In serious cases, a psychiatrist should be consulted. This is consistent with the core concept of the integrated medical-nursing-patient care model. The results of this study showed that the SAS and SDS scores of the observation group after the intervention were lower than those of the preintervention and control groups (*p* < 0.05), and the compliance and satisfaction with care were higher than those of the control group (*p* < 0.05). This can facilitate a smooth transition from hospital care to home care, alleviate the guilt and self-blame of parents, reduce parents' anxiety and psychological pressure, create conditions for establishing a good doctor-patient relationship and parent-child relationship, and reduce the occurrence of medical disputes [10].

RETRACTED

## 8. Conclusion

To summarize, the clinical application of the integrated medical-nurse-patient care model in children with CEA is effective. It effectively reduced the complication rate and postoperative readmission rate of CEA and the number of unnecessary hospital visits, detecting and intervening in postoperative complications early. It also effectively improved the negative psychological state of parents, increasing compliance and satisfaction, and is a more ideal model for CEA care. It is an ideal model of CEA care and worthy of clinical promotion. Currently, the integrated healthcare model is widely used in clinical care, but few studies have discussed the difficulties and obstacles in its implementation, as well as its solutions. Second, the implementation of the integrated healthcare model requires the concerted effort of all healthcare professionals to study and develop a uniform and standardized workflow and specific implementation methods. Although the healthcare integration model has been carried out for many years, the specific implementation and evaluation methods vary from hospital to hospital, and there is variability among hospitals of different levels and fields, so there is still a need to explore a more reasonable healthcare integration model [13–20].

## Figures and Tables

**Figure 1:** Attention-LSTM model.

**Figure 2:** NFM model.

**Figure 3:** Percentage increase in hospital admissions for respiratory diseases per 10 *μ*g increase in each pollutant concentration (95% CI, red means statistically significant).

**Figure 4:** Percentage increase in hospital admissions for circulatory disease per 10 *μ*g increase in each pollutant concentration (95% CI, red represents statistical significance).

**Figure 5:** Percentage increase in hospital admissions.

**Table 1:** Comparison of general information of children in two groups.

Project	Control group (*n* = 60)	Observation group (*n* = 60)	*x* ^2^/*t*	*P* value
Gender (male/female) (example)	38/22	41/19	0.333	0.564
Gestational age at birth (W, $\bar{x}\pm s$)	38.4 ± 5.68	38.9 ± 4.63	−0.515	0.608
Birth weight (kg, $\bar{x}\pm s$)	2.72 ± 0.24	2.84 ± 0.53	−1.898	0.113
1-minute Apgar score (points, $\bar{x}\pm s$)	9 ± 0.35	9 ± 0.28	<0.001	1.000
Father's age (years, $\bar{x}\pm s$)	27.73 ± 5.27	26.82 ± 4.5	0.867	0.358
Mother's age (years, $\bar{x}\pm s$)	25.23 ± 6.25	24.18 ± 6.74	1.006	0.675
Education level (example)				
College degree or above	37	42		
High school	18	14		
Junior middle school	5	4		

RETRACTED

**Table 2:** Comparison of the abnormalities found in the two groups of children after surgery.

Group	Number of cases	Number of revisits	Rehospitalization rate (person (%))	1-hour visit rate of children with suspected postoperative complications (person (%))	Accuracy rate of children with suspected postoperative complications (person (%))
Observation group	60	18	17 (28.33)	15 (88.33)	16 (88.89)
Control group	60	39	28(46.67)	9(23.07)	25(64.10)
*x* ^2^ value			4.302	-	-
*P* value			0.038	<0.001	0.048

**Table 3:** Comparison of SAS and SDS scores before and after intervention for parents of children in both groups (scores, $\bar{x}\pm s$).

Group	Number of cases	SAS score		SDS score	
		Before intervention	After intervention	Before intervention	After intervention
Observation group	60	65.41 ± 4.26	40.15 ± 3.14	61.31 ± 4.17	41.73 ± 2.57
Control group	60	64.37 ± 3.85	58.27 ± 3.18	60.89 ± 4.59	54.41 ± 3.72
t value		1.403	−31.407	0.525	−21.723
*P* value		0.163	<0.001	0.601	<0.001

**Table 4:** Comparison of compliance (%).

Group	Number of cases	Noncompliance	Partial compliance	Complete compliance	Compliance rate	*x* ^2^ value	*P* value
Observation group	60	1 (1.67)	2 (3.33)	57 (95.00)	59 (98.330)	4.821	0.028
Control group	60	7 (6.67)	6 (10.00)	47 (78.33)	53 (88.33)		

**Table 5:** Percentage increase in hospital admissions (95% CI) for three systemic disease categories per 10 *μ*g increase in each pollutant concentration (0.1 mg increase in CO).

Contaminants	Respiratory hospitalization	Circulatory system hospitalization	Digestive system hospitalization
*PM*_2.5_	0.3 (0.04, 0.57)^*∗*^	0.24 (−0.1, 0.59)	0.03 (−0.3, 0.36)
*PM*_10_	0.21 (0.04, 0.39)^*∗*^	0.21 (−0.01, 0.43)	0.04 (−0.16, 0.25)
*SO*_2_	2.43 (0.63, 4.26)^*∗*^	2.84 (0.58, 5.16)^*∗*^	0.46 (−1.62, 2.58)
*NO*_2_	1.17 (0.57, 1.77)^*∗*^	1.4 (0.65, 2.16)^*∗*^	0.67 (−0.03, 1.38)
CO	0.47 (0.16, 0.78)^*∗*^	0.6 (0.21, 0.99)^*∗*^	0.27 (−0.1, 0.64)
*O*_3_	0.16 (0.55, 0.22)	−0.18 (−0.64, 0.28)	−0.12 (−0.54, 0.31)

^*∗*^ *p* < 0.05, statistically significant; all pollutant concentrations are same-day concentrations (lag0).

## Data Availability

The datasets used and analyzed during the current study are available from the corresponding author upon reasonable request.

RETRACTED

## References

[1] Vinales J. J. (2013). Evaluation of Makaton in practice by children’s nursing students. *Nursing Children and Young People*.

[2] Raitio A., Cresner R., Smith R., Jones M. O., Losty P. D. (2016). Fluoroscopic balloon dilatation for anastomotic strictures in patients with esophageal atresia: a fifteen-year single centre UK experience. *Journal of Pediatric Surgery*.

[3] Blodgett T., Fawcett J., DeSanto-Madeya S. (2017). *A Book Review of Contemporary Nursing Knowledge: Analysis and Evaluation of Nursing Models and Theories, Nursing Science Quarterly*.

[4] Zhang C., Xie T., Yang K. (2019). Positioning optimisation based on particle quality prediction in wireless sensor networks. *IET Networks*.

[5] Alisa H. (2001). Long-gap oesophageal atresia: a nursing perspective[J]. *Journal of Child Health Care for Professionals Working with Children in the Hospital & Community*.

[6] Krishnan U., Mousa H., Dall’Oglio L. (2016). ESPGHAN-NASPGHAN guidelines for the evaluation and treatment of gastrointestinal and nutritional complications in children with esophageal atresia-tracheoesophageal fistula. *Journal of Pediatric Gastroenterology and Nutrition*.

[7] Lebœuf M., Cortes D., Hocquemiller R. (2017). Quality of life after surgical treatment for esophageal atresia: long-term outcome of 154 patients. *European Journal of Pediatric Surgery*.

[8] Linde K., Streng A., Hoppe A. (2006). The programme for the evaluation of patient care with acupuncture (PEP-Ac) - a project sponsored by ten German social health insurance funds. *Acupuncture in Medicine*.

[9] Lin H.-Y., Lin S.-P., Lin H.-Y. (2012). Functional independence of Taiwanese children with VACTERL association. *American Journal of Medical Genetics, Part A*.

[10] Rozas-García M. R., Costa J., Francés L., Viñas-Llebot H., Paulí A., Martínez C. (2008). Autoevaluación del aprendizaje en enfermería con ejercicios interactivos del programa Hot Potatoes. *Revista de la Fundación Educación Médica*.

[11] Mastiliaková D., Gibbs A., Adamczyk R. (2013). Evaluation OF learning outcomes for critical thinking in a nursing study programme. *University Review*.

[12] Aite L., Bevilacqua F., Zaccara A. (2016). Seeing their children in pain: symptoms of posttraumatic stress disorder in mothers of children with an anomaly requiring surgery at birth. *American Journal of Perinatology*.

